This article has been retracted.

# BCORL1 is an independent prognostic marker and contributes to cell migration and invasion in human hepatocellular carcinoma

**DOI:** 10.1186/s12885-016-2154-z

**Published:** 2016-02-15

**Authors:** Guozhi Yin, Zhikui Liu, Yufeng Wang, Changwei Dou, Chao Li, Wei Yang, Yingmin Yao, Qingguang Liu, Kangsheng Tu

**Affiliations:** Department of Hepatobiliary Surgery, the First Affiliated Hospital of Xi’an Jiaotong University, No.277 Yanta West Road, Xi’an, 710061 China

**Keywords:** BCL6 corepressor-like 1, Hepatocellular carcinoma, Prognostic marker, E-cadherin, Tumor metastasis

## Abstract

**Background:**

The deregulation of E-cadherin has been considered as a leading cause of hepatocellular carcinoma (HCC) metastasis. BCL6 corepressor-like 1 (BCORL1) is a transcriptional corepressor and contributes to the repression of E-cadherin. However, the clinical significance of BCORL1 and its role in the metastasis of HCC remain unknown.

**Methods:**

Differentially expressed BCORL1 between HCC and matched tumor-adjacent tissues, HCC cell lines and normal hepatic cell line were detected by Western blot. The expression of BCORL1 was altered by siRNAs or lentivirus-mediated vectors. Transwell assays were performed to determine HCC cell invasion and migration.

**Results:**

Increased expression of BCORL1 protein was detected in HCC specimens and cell lines. Clinical association analysis showed that BCORL1 protein was expressed at significant higher levels in HCC patients with multiple tumor nodes, venous infiltration and advanced TNM tumor stage. Survival analysis indicated that high expression of BCORL1 protein conferred shorter overall survival (OS) and recurrence-free survival (RFS) of HCC patients. Multivariate Cox regression analysis disclosed that BCORL1 expression was an independent prognostic marker for predicting survival of HCC patients. Our in vitro studies demonstrated that BCORL1 prominently promoted HCC cell migration and invasion. Otherwise, an inverse correlation between BCORL1 and E-cadherin expression was observed in HCC tissues. BCORL1 inversely regulated E-cadherin abundance and subsequently facilitated epithelial-mesenchymal transition (EMT) in HCC cells. Notably, the effect of BCORL1 knockdown on HCC cells was abrogated by E-cadherin silencing.

**Conclusions:**

BCORL1 may be a novel prognostic factor and promotes cell migration and invasion through E-cadherin repression-induced EMT in HCC.

**Electronic supplementary material:**

The online version of this article (doi:10.1186/s12885-016-2154-z) contains supplementary material, which is available to authorized users.

## Background

Hepatocellular carcinoma (HCC) is the 5th most frequent malignancy and 3rd most common cause of cancer mortality in the world [1]. Due to high infection rate of hepatitis B virus (HBV), HCC has been considered as a serious health problem in China [2]. Postoperative recurrence and metastasis is the leading cause of poor prognosis for HCC patients [3]. E-cadherin, an important member of cadherin family, functions as a key factor in regulation of epithelial cell-to-cell adhesion [4]. Numerous studies have reported that impaired expression and/or dysfunction of E-cadherin leads to loss of epithelial phenotype and promotes cell migration and invasion in human cancer [5]. Furthermore, loss expression of E-cadherin contributes to epithelial-mesenchymal transition (EMT), which is a main cause of tumor metastasis [6]. It has been demonstrated that reduced expression of E-cadherin was correlated with invasion and metastasis of various human cancers including HCC [7]. Mechanistically, transcriptional repressors including Snail, Slug, Twist, Zinc finger E-box-binding homeobox 1/2 (ZEB1/2) and C-terminal-binding protein (CtBP) are involved in the regulation of E-cadherin expression [8, 9].

BCL6 corepressor-like 1 (BCORL1) is a recently identified transcriptional corepressor [10]. Co-immunoprecipitation indicates that BCORL1 interacts with class II histone deacetylases, such as HDAC4, HDAC5 and HDAC7 [10]. Furthermore, BCORL1 represses the expression of E-cadherin via locating on the E-cadherin promoter. Otherwise, BCORL1 interacts with the amino terminus of CtBP via the PXDLS motif and suppresses the transcription of E-cadherin [10]. It is conceivable, therefore, that BCORL1 might promote tumor metastasis. Yasushi Totoki et al. validated that BCORL1- E74-like factor 4 (ELF4) was a somatic fusion transcripts generated by rearrangements through sequencing analysis of the HCC and matched non-cancerous liver tissues [11]. Compared with the expression of wild-type BCORL1 and ELF4 gene in non-tumor tissues, increased expression of fusion transcripts was confirmed in HCC tissues by quantitative reverse transcription-PCR (qRT-PCR) [11]. However, in HCC, the clinical significance of BCORL1 and its functional role remain poorly investigated.

This study confirms that increased expression of BCORL1 is observed in HCC tissues and cell lines. Elevated expression of BCORL1 is evidently associated with poor prognostic features and reduced survival of HCC patients. BCORL1 promotes the invasive behavior of HCC cells and inversely regulates the abundance of E-cadherin in HCC cells. Mechanistically, our data indicate that BCORL1 promotes the invasive ability of HCC cells by suppressing E-cadherin and subsequently facilitating EMT.

## Methods

### Cell culture and transfection

Human HCC cells (HepG2, Hep3B, HCCLM3 and MHCC97H) and immortalized liver cell line (LO2) were obtained from the Institute of Biochemistry and Cell Biology, Chinese Academy of Science, China. Cells were maintained in Dulbecco’s Modified Eagle Medium (DMEM, Gibco, Grand Island, NY, USA), which was supplemented with 10 % fetal bovine serum (FBS, Gibco), 100 μg/ml penicillin, and 100 μg/ml streptomycin (Sigma, St-Louis, MO, USA), at 37 °C in a 5 % CO_2_ incubator.

A specific BCORL1 siRNA (5′-AGC CCU CAG CCU CUG CCA CG-3′), E-cadherin siRNA (5′-CAG ACA AAG ACC AGG ACU A-3′) and a nonspecific duplex oligonucleotide as a negative control were synthesized by Sangon Biotech (Shanghai) Co., Ltd. (Shanghai, China). A predesigned siRNA directed against human BCORL1 (BCORL1 siRNA-1) was purchased from Qiagen (SI00311437; Shanghai, China). The siRNAs mentioned above were transfected into HCC cells using Lipofectamine 2000 following the manufacturer’s instructions (Invitrogen, Carlsbad, CA, USA). ORF lentiviral expression clone (EX-W1876-Lv105-5) for BCORL1 was purchased from Genecopoeia (Guangzhou, China). Lentivirus packaging and transduction were performed using Lenti-Pac HIV Expression Packaging Kit (HPK-LvTR-20, Genecopoeia) following manufacturer’s instructions.

### In vitro migration, invasion and BrdU incorporation assays

The migration and invasion of HCC cells were measured using 24-well Transwell plates (8-μm pore size, Corning, NY, USA) as previously described [12]. For migration assays, 5 × 10^4^ cells were suspended in 200 μL serum reduced DMEM medium and added into the upper chamber with a non-coated membrane. For invasion assays, chamber inserts were coated with Matrigel (BD Biosciences, Franklin Lakes, NJ, USA) at 1:7 dilutions. For the proliferation assay, HCC cells were seeded into 96-well plates at 5000 cells per well for 24 h and assessed using a Cell Proliferation ELISA, BrdU (5-bromodeoxyuridine) (chemiluminescent) (Roche, USA) as previously described [13].

### Patients and follow-up

HCC specimens and matched tumor-adjacent tissues were obtained from 86 adult patients, who underwent surgical resection of primary HCC between 2006 and 2008 at the First Affiliated Hospital of Xi’an Jiaotong University. All samples were used after obtaining informed consent. Patients that met the following criteria were included: (a) confirmed pathologic diagnosis, (b) no preoperative chemotherapy or radiotherapy, (c) no distant metastases, (d) curative liver resection, and (e) complete clinical-pathologic and follow-up data. Tumor differentiation level was assessed using Edmondson-Steiner grading. The TNM stage of HCC was determined based on the guide of the 6th International Union Against Cancer/American Joint Committee on Cancer (UICC/AJCC). The clinicopathological data are shown in Table 1.

**Table 1:** Clinicopathological correlation of BCORL1 expression in HCC

Clinicopathologic features		n	BCORL1		*P*
			High expression (*n* = 43)	Low expression (*n* = 43)	
Age (y)	≤50	34	20	14	0.186
	>50	52	23	29	
Sex	Male	76	37	39	0.501
	Female	10	6	4	
HBsAg	No	12	7	5	0.534
	Yes	74	36	38	
Serum AFP level (ng/mL)	≤20	26	14	12	0.639
	>20	60	29	31	
Tumor size (cm)	≤5	39	18	21	0.516
	>5	47	25	22	
No. of tumor nodules	1	71	31	40	0.011*
	≥2	15	12	3	
Cirrhosis	Absent	20	7	13	0.126
	Present	66	36	30	
Venous infiltration	Absent	41	15	26	0.018*
	Present	45	28	17	
Edmondson-Steiner grading	I+II	65	30	35	0.209
	III+IV	21	13	8	
TNM tumor stage	I+II	64	28	36	0.048*
	III+IV	22	15	7	

*HCC* hepatocellular carcinoma, *HBV* hepatitis B virus, *AFP* alpha-fetoprotein, *TNM* tumor-node-metastasis. *Statistically significant

The follow-up data were collected by the end of December 2013 (with a median follow-up time of 35.5 months). Primary endpoints included the time to recurrence and overall survival. The date of resection to the date of tumor recurrence diagnosis was defined as the time to recurrence. The duration between the date of resection and the date of death or last follow-up was calculated as the overall survival. This study was approved by the Ethics Committee of the Xi’an Jiaotong University.

### qRT-PCR

qPCR primer against to Homo sapiens E-cadherin (NM_004360.2; HQP023466) and GAPDH (NM_002046.3; HQP006940) were purchased from Genecopoeia (Guangzhou, China). The PCR amplification of the E-cadherin and GAPDH mRNAs was performed according the instruction of ABI PRISM 7300 Sequence Detection System (Applied Biosystems, Foster City, CA, USA) and the SYBR^®^ Premix Ex Taq™ ii (Perfect Real Time) Kit (Takara Bio, Shiga, Japan), as previous described [14].

### Western blot analysis

Proteins from lysed cells were separated by sodium dodecyl sulfate polyacrylamide gel electrophoresis (SDS-PAGE) and transferred to nitrocellulose membranes (Bio-Rad, Hercules, CA, USA). Nonspecific binding sites were blocked with 5 % BSA in TBST for 60 min at room temperature. Blots were incubated with BCORL1 (PA5-24333, Thermo Fisher Scientific Pierce, Waltham, MA, USA), E-cadherin (24E10, #3195; Cell Signaling, Beverly, MA, USA) or GAPDH (G8140; US Biological, Swampscott, MA, USA) antibodies overnight at 4 °C. The membranes were then incubated with horseradish peroxidase (HRP)-conjugated sheep anti-mouse or donkey anti-rabbit secondary antibodies (Bio-Rad, Hercules, CA, USA) diluted at 1:10000, and detected using the Western Blotting Luminol Reagent (sc-2048, Santa Cruz, CA, USA) [15].

### Immunohistochemical staining

Paraformaldehyde-fixed paraffin sections were used to perform the immunohistochemistry. BCORL1 (Thermo Fisher Scientific Pierce) and E-cadherin (Cell Signaling) antibodies at a dilution 1:100 were used in immunohistochemistry with streptavidin peroxidase conjugated (SP-IHC) method. Detailed procedures of immunohistochemistry were performed as previous reported [16]. The percentage of positive tumor cells was scored according to the following criteria: 0, less than 10 %; 1, 10–30 %; 2, 31–50 %; 3, more than 50 %.

### Immunofluorescence

The primary E-cadherin antibody (Cell Signaling) was used in the immunofluorescence assays. The secondary antibody was an Alexa Fluor–conjugated IgG (Invitrogen, Carlsbad, CA, USA). Immunofluorescence was performed as previous reported [15].

### Statistical analysis

All statistical analyses were performed using the SPSS statistical package for Windows Version 13 (SPSS, Chicago, IL, USA) or GraphPad Prism 5 software (GraphPad Software, Inc, San Diego, CA, USA). The quantitative data were compared between groups using the Student’s *t*-test or ANOVA. Categorical data were analyzed using the Pearson chi-squared test. The Kaplan-Meier method and log-rank test were used to compare the cumulative recurrence and survival rates. The independent factors influencing the survival and recurrence of HCC patients were determined using the Cox proportional hazards model. Correlation analysis was tested by the Pearson’s correlation coefficient. A value of *P* < 0.05 was considered to be statistically significant.

## Results

### Expression of BCORL1 in clinical specimens and HCC cells

Initially, 86 pairs of HCC tissues and matched noncancerous tissues were subjected to immunoblotting to detect the protein level of BCORL1. As indicated in Fig. 1a, the level of BCORL1 protein in HCC tissues was significantly higher as compared with that in matched tumor-adjacent tissues (*P* < 0.05). Furthermore, the expression of BCORL1 protein was determined by Western blot in a normal hepatic cell line (LO2) and a panel of HCC cell lines (HepG2, Hep3B, MHCC97H and HCCLM3). Our data disclosed that BCORL1 protein levels in HCC cell lines were significantly up-regulated compared with that in LO2 (*P* < 0.05, Fig. 1b). Otherwise, the levels of BCORL1 protein in HCC cell lines (MHCC97H and HCCLM3) with high metastatic ability were evidently higher than those in HCC cell lines (HepG2 and Hep3B) with low metastatic ability (*P* < 0.05, Fig. 1b). On the contrary, E-cadherin mRNA was expressed at a significant lower level in HCC cell lines, especially in high invasive cell lines (*P* < 0.05, Fig. 1c). Therefore, our results indicate that BCORL1 is overexpressed in HCC specimens and cell lines.

**Fig. 1:** BCORL1 is abnormally up-regulated in human HCC. **a** Representative Western blot analysis showed the expression of BCORL1 in the HCC (T) and matched nontumor tissues (NT). Quantitative analysis indicated that BCORL1 protein was significantly up-regulated in HCC tissues as compared with that in nontumor tissues. *n* = 86; ^*^ *P* < 0.05 by *t* test. **b** The expression levels of BCORL1 protein in HCC cell lines (HepG2, Hep3B, MHCC97H and HCCLM3) and a normal hepatic cell line (LO2). *n* = 3; ^*^ *P* < 0.05 by ANOVA. **c** The expression levels of E-cadherin mRNA in HCC cell lines and a normal hepatic cell line. *n* = 3; ^*^ *P* < 0.05 by ANOVA

### Clinical significance of BCORL1 expression in HCC cases

The expression of BCORL1 was divided into low expression group (*n* = 43) and high expression group (*n* = 43) based on its cutoff value, which was defined as the median value of the cohort of patients tested. The correlation between the expression of BCORL1 and clinicopathologic features of HCC patients was summarized in Table 1. By statistical analysis, increased level of BCORL1 was significantly correlated with multiple tumor nodes (*P* = 0.011), venous infiltration (*P* = 0.018) and advanced tumor-node-metastasis (TNM) tumor stage (*P* = 0.048). Next, we evaluated the prognostic value of BCORL1 expression in HCC patients through Kaplan-Meier survival analysis. HCC patients with high expression of BCORL1 had an obviously reduced 5-year overall survival (OS) as compared with those with low expression of BCORL1 (*P* = 0.002, Fig. 2). Furthermore, it was showed that high expression of BCORL1 was associated with shorter recurrence-free survival (RFS) (*P* = 0.001, Fig. 2). In addition, BCORL1 expression was indicated to be an independent predictor of 5-year OS and RFS of HCC patients (*P* = 0.002 and *P* = 0.003, Table 2) through multivariate Cox regression analysis. Thus, our data demonstrate that BCORL1 is a potential valuable prognostic indicator for the prognosis of HCC patients.

**Fig. 2:** Prognostic value of BCORL1 for HCC patients. Kaplan-Meier overall survival (OS) and recurrence-free survival (RFS) curves of HCC patients in accordance with their expression status of BCORL1 protein. High expression of BCORL1 protein conferred a worse 5-year OS and RFS for HCC patients. The expression of BCORL1 was divided into low level group (*n* = 43) and high level group (*n* = 43) based on the cutoff value which was defined as the median protein level of the 86 HCC samples detected by Western blot

**Table 2:** Multivariate Cox regression analysis of 5-year OS and RFS of 86 HCC patients

Variables	OS			RFS		
	HR	95 % CI	*P*	HR	95 % CI	*P*
No. of tumor nodules (1 *vs* ≥2)	0.736	0.578–0.939	0.014*	0.753	0.588–0.965	0.025*
Venous infiltration (Absent *vs* Present)	0.812	0.646–1.022	0.076	0.796	0.632–1.004	0.054
TNM tumor stage (I+II *vs* III+IV)	0.267	0.194–0.367	<0.001*	0.236	0.170–0.328	<0.001*
BCORL1 expression (Low *vs* High)	0.660	0.509–0.854	0.002*	0.672	0.518–0.872	0.003*

*OS* overall survival, *RFS* recurrence-free survival, *TNM* tumor-node-metastasis, *HR* hazard ratio, *CI* confidence interval. *Statistically significant

### BCORL1 promotes cell migration and invasion in HCC cells

To further elucidate the biological function of BCORL1 in HCC, specific siRNAs targeting BCORL1 were used for loss-of-function experiments in HCCLM3 cells. As confirmed by Western blot, the expression of BCORL1 protein was significantly down-regulated by BCORL1 siRNA in HCCLM3 cells compared to control cells (*P* < 0.05, Fig. 3a and Additional file 1: Figure S1A). Transwell migration assays were performed to test the effect of BCORL1 knockdown on tumor cell migration. BCORL1 knockdown significantly reduced the migratory ability of HCCLM3 cells (*P* < 0.05, Fig. 3b and Additional file 1: Figure S1B). Furthermore, as determined by Transwell invasion assays, the invasion of HCCLM3 cells was prominently decreased after BCORL1 knockdown in HCCLM3 cells (*P* < 0.05, Fig. 3b and Additional file 1: Figure S1B). Similarly, BCORL1 knockdown evidently suppressed cell migration and invasion in MHCC97H cells (*P* < 0.05, respectively). However, BCORL1 knockdown did not evidently influence cell proliferation in both MHCC97H and HCCLM3 cells as assessed by BrdU incorporation assays (*P* = 0.102 and *P* = 0.120, respectively, Additional file 2: Figure S2). Next, BCORL1 overexpressing Hep3B cells were established by lentivirus-mediated transfection and confirmed by immunoblotting (*P* < 0.05, Fig. 3c). In contrast, BCORL1 overexpression facilitated the migration and invasion of Hep3B cells (*P* < 0.05, respectively, Fig. 3d). Thus, these results indicate that BCORL1 truly promotes the metastatic behaviors of HCC cells in vitro.

**Fig. 3:** BCORL1 increases migrated and invaded HCC cells. **a** HCCLM3 cells with BCORL1 siRNA and scrambled siRNA transfection, respectively, were subjected to immunoblotting for BCORL1. *n* = 6; ^*^ *P* < 0.05 by *t* test. **b** Transwell migration assays showed that BCORL1 knockdown inhibited cell migration in HCCLM3 cells. As assessed by Transwell invasion assays, HCCLM3 cell invasion was inhibited by BCORL1 knockdown. ^*^ *P* < 0.05 by *t* test; *n* = 3. **c** Hep3B cells that were infected with BCORL1 or empty vector (EV) lentiviruses, were detected by Western blot. *n* = 6; ^*^ *P* < 0.05 by *t* test. **d** BCORL1 overexpression increased the number of migrated and invaded cells as measured by Transwell assays in Hep3B cells. ^*^ *P* < 0.05 by *t* test; *n* = 3

### BCORL1 inversely regulates E-cadherin abundance in HCC

Further studies were performed to disclose the molecular mechanisms by which BCORL1 promoted HCC cell migration and invasion. Previous studies reported that BCORL1 acted as a transcriptional corepressor and repressed the expression of E-cadherin, which was considered as an EMT-related epithelial marker and inhibited cancer cell migration and invasion [8, 10]. The expressions of BCORL1 and E-cadherin were further detected by immunohistochemistry in serial sections of 86 HCC cases. Based on the immunohistochemical score, the immunoreactivity of E-cadherin and BCORL1 was considered as either negative (score 0) or positive (scores 1–3). Positive expression of E-cadherin was detected in 70.0 % (21/30) of the HCC specimens with negative expression of BCORL1, whereas only 35.7 % (20/56) of BCORL1 positively expressing HCC cases showed a positive E-cadherin signal (*P* < 0.05, Fig. 4a). Otherwise, Pearson’s correlation analysis confirmed that BCORL1 expression was inversely correlated with E-cadherin in HCC tissues (*r* = −0.723, *P* = 0.002, Fig. 4b). Furthermore, HCCLM3 cells that were transfected with BCORL1 siRNA or scrambled siRNA were subjected to qRT-PCR and Western blot for E-cadherin. Our data found that BCORL1 knockdown resulted in obvious increase of E-cadherin expression in HCC cells (*P* < 0.05, respectively, Fig. 4c and 4d). On the contrary, BCORL1 overexpression significantly reduced E-cadherin expression in Hep3B cells (*P* < 0.05, respectively, Fig. 4e and 4f). Furthermore, the regulatory effect of BCORL1 on E-cadherin expression was further confirmed by immunofluorescence (Fig. 5). Interestingly, BCORL1 knockdown decreased the levels of vimentin and N-cadherin, two EMT-related mesenchymal markers, in HCCLM3 cells (*P* < 0.05, respectively, Fig. 4d), while BCORL1 overexpression increased the expressions of vimentin and N-cadherin in Hep3B cells (*P* < 0.05, respectively, Fig. 4f), indicating BCORL1 affected EMT in HCC cells. Thus, BCORL1 inversely regulates E-cadherin abundance and facilitates EMT in HCC.

**Fig. 4:** BCORL1 is inversely correlated with E-cadherin in HCC. **a** The positive expression rate of E-cadherin in BCORL1 positive HCC specimens was significantly lower than that in BCORL1 negative cases. ^*^ *P* < 0.05 by Pearson chi-squared test. **b** Representative immunohistochemical staining showed weak staining of E-cadherin (III) in BCORL1 positive-expressing tumor (I) and strong staining of E-cadherin (IV) in BCORL1 negative-expressing tumor (II). Scale bar: 50 μm. **c** qRT-PCR analysis of E-cadherin mRNA expression in HCCLM3 cells with BCORL1 siRNA or scrambled siRNA transfection. ^*^ *P* < 0.05 by *t* test, *n* = 3. **d** BCORL1 knockdown increased the level of E-cadherin protein and reduced the expression of vimentin and N-cadherin in HCCLM3 cells. ^*^ *P* < 0.05 by *t* test, *n* = 6. **e** qRT-PCR analysis of E-cadherin mRNA expression in Hep3B cells with BCORL1or empty vector (EV) lentiviruses infection. ^*^ *P* < 0.05 by *t* test, *n* = 3. **f** BCORL1 overexpression decreased the level of E-cadherin protein and up-regulated the expression of vimentin and N-cadherin in Hep3B cells. ^*^ *P* < 0.05 by *t* test, *n* = 6

**Fig. 5:** Immunofluorescent staining of E-cadherin in HCC cells. HCC cells that were treated with corresponding vectors were subjected to immunofluorescence for E-cadherin. BCORL1 knockdown increased E-cadherin immunofluorescence densities in HCCLM3 cells and BCORL1 overexpression reduced the expression of E-cadherin in Hep3B cells. DAPI stain (blue) was used to identify nuclei. Scale bar: 20 μm

### BCORL1 promotes the migration and invasion of HCC cells by suppressing E-cadherin

To validate whether E-cadherin participates in the promoting effects of BCORL1 on HCC cell migration and invasion, BCORL1 down-regulating HCCLM3 cells were subsequently transfected with scrambled siRNA or E-cadherin siRNA. E-cadherin knockdown was confirmed by Western blot (*P* < 0.05, Fig. 6a). Transwell assays indicated that E-cadherin knockdown abolished the inhibitory effect of BCORL1 knockdown on the mobility of HCCLM3 cells, resulting in a significant increase of migrated and invaded cell numbers (*P* < 0.05, Fig. 6b). Taken together, these results suggest that E-cadherin probably acts as a downstream factor of BCORL1 and mediates the contributing effects of BCORL1 on HCC cell migration and invasion.

**Fig. 6:** E-cadherin knockdown abolishes the anti-metastatic effect of BCORL1 knockdown. **a** Scrambled siRNA or E-cadherin siRNA was transfected into BCORL1 down-regulating HCCLM3 cells and confirmed by Western blot. *n* = 6; ^*^ *P* < 0.05 by *t* test. **b** E-cadherin knockdown increased cell migration and invasion in BCORL1 down-regulating HCCLM3 cells. *n* = 3, ^*^ *P* < 0.05 by *t* test

## Discussion

The expression of BCORL1 was highest in testis and prostate tissues, medium in lymphocytes and spleen, and low in many other tissues as demonstrated by Northern blot assay [10]. Previous study has reported that the expression of BCORL1-ELF4 chimeric transcript in HCC tissues is obviously higher than the expression of wild-type BCORL1 and ELF4 mRNA in noncancerous liver tissues [11]. However, the expression status of BCORL1 protein in HCC specimens and its clinical significance are largely unknown. In this study, we initially detected the expression of BCORL1 protein in HCC tissues and matched tumor-adjacent tissues. Our data found that BCORL1 protein in tumor tissues was significantly increased as compared with that in nontumor tissues. Furthermore, elevated expression of BCORL1 protein was observed in HCC cell lines, especially in those with highly metastatic ability (HCCLM3 and MHCC97H). While the expression of E-cadherin mRNA showed an opposite pattern in HCC cell lines. Clinical association analysis indicated that high expression of BCORL1 protein was correlated with poor clinical features of HCC including multiple tumor nodes, venous infiltration and advanced TNM tumor stage. These data suggest that BCORL1 may function as an oncogene and contributes to tumor metastasis in HCC. Notably, survival analysis demonstrated that high expression of BCORL1 conferred significant shorter 5-year OS and RFS of HCC patients. Consistent with our data, patients with up-regulation of BCORL1 mRNA have a shorter median overall survival (33.02 months *vs* control: 45.07 months) and recurrence-free survival (8.64 months *vs* control: 19.65 months) in the cBioPortal for Cancer Genomics data, though the difference had no statistical significance [17, 18]. Moreover, Multivariate Cox repression analysis disclosed that BCORL1was an independent predictor of the prognosis of HCC patients. The mechanism by which BCORL1 is regulated in cancer is poorly investigated. Data analysis with the gene expression microarray showed that BCORL1 was a potential target gene of miR-155 in the azoxymethane (AOM) and dextran sulfate sodium (DSS) induced colitis-associated colon cancer mouse model [19]. Thus, it is worth to disclose the mechanism by which BCORL1 is up-regulated in HCC. Taken together, our data indicate that BCORL1 expression is important for the survival prediction of HCC patients.

Mutations of *BCORL1* have been found in acute myelogenous leukemia, myelodysplastic syndromes and intracranial germ cell tumours [20–24]. Furthermore, *BCORL1* is a tumor suppressor gene that may be inactivated by mutations in acute myeloid leukemia [21]. While BCORL1 expression is not a predisposing factor of familial breast cancer [25]. However, studies about the biological function of BCORL1 in human cancers are rarely reported. According to our clinical research, we evaluated the influence of BCORL1 alteration on the migration and invasion of HCC cells. As expected, BCORL1 knockdown prominently reduced the migratory and invasive abilities of HCC cells. Otherwise, BCORL1 overexpression significantly promoted HCC cell migration and invasion. However, what is the underlying mechanism involved in the pro-metastatic role of BCORL1 in HCC? Pagan JK et al. have shown that BCORL1 mediates the repression of E-cadherin, which is critical to maintain normal epithelial cell contact and its downregulation has been seen in the majority of human cancers including HCC [4, 10, 26]. Decreased expression of E-cadherin is considered as the initiation of the EMT, which plays important role in the spread of malignant hepatocytes during HCC progression [27]. Thus, we investigated the regulatory effect of BCORL1 on the expression of E-cadherin. In HCC specimens, the expressions of E-cadherin in BCORL1 positive cases were prominently lower than those in BCORL1 negative cases. Furthermore, an inverse correlation between BCORL1 and E-cadherin expression in HCC tissues was confirmed by the immunohistochemical experiments. Our in vitro studies demonstrated that BCORL1 knockdown significantly increased the mRNA and protein levels of E-cadherin in HCCLM3 cells. On the contrary, BCORL1 overexpression reduced E-cadherin expression in Hep3B cells. Importantly, BCORL1 positively regulated the abundance of vimentin and N-cadherin, which were considered as mesenchymal markers in EMT, in HCC cells. These results indicate that BCORL1 may be a novel regulator of EMT in HCC. Moreover, E-cadherin knockdown abrogated BCORL1 deletion-induced suppression of HCC cell migration and invasion. Since BCORL1 was reported as corepressor on E-cadherin promoter [10]. A number of transcriptional repressors are known to regulate E-cadherin expression, including Snail [28], Slug [29], Twist [30], and ZEB/δEF1 [31, 32], and it is possible that BCORL1 might function together with these repressors, or as part of a separate as yet unknown complex [10]. Thus, these data suggest that BCORL1 may promote the migratory and metastatic ability of HCC cells by repressing the expression of E-cadherin and subsequently promoting EMT.

In conclusion, this study confirms the overexpression of BCORL1 in HCC. And increased expression of BCORL1 is associated with poor prognostic features. We demonstrate that BCORL1 expression is an independent prognostic marker for HCC patients. Our in vitro experiments reveal that BCORL1 promotes the migration and invasion of HCC cells. Furthermore, BCORL1 inversely regulates E-cadherin abundance and promotes EMT in HCC cells. Altogether, deregulation of BCORL1 may play a fundamental role in tumor metastasis and may serve as a novel prognostic indicator and potential therapeutic target for HCC.

## Conclusions

In summary, this study shows that the expression of BCORL1 is up-regulated in HCC tissues as compared with that in matched adjacent noncancerous tissues. Furthermore, the relative expression of BCORL1 in HCC cell lines is significantly higher than that in the normal hepatic cell line. Clinical association analyses indicate that high expression of BCORL1 is evidently associated with poor prognostic features of HCC. Notably, BCORL1 expression is an independent prognostic marker for predicting 5-year OS and RFS of HCC patients. In vitro studies demonstrate that BCORL1 knockdown inhibits cell migration and invasion in HCCLM3 cells. In contrast, BCORL1 overexpression increases the number of migrated and invaded Hep3B cells. Interestingly, BCORL1 is inversely correlated with the levels of E-cadherin in HCC tissues. Otherwise, our data indicate that BCORL1 inversely regulates the abundance of E-cadherin and subsequently facilitates EMT in HCC cells. Importantly, E-cadherin knockdown abrogates the effects of BCORL1 knockdown on inhibiting HCC cell mobility. This study reveals that BCORL1 may play a critical role in the tumor metastasis of HCC by suppressing E-cadherin and may be a potential prognostic biomarker and therapeutic target for HCC.

## Additional files

Additional file 1: Figure S1. BCORL1 knockdown inhibits cell migration and invasion in HCCLM3 cells. A) HCCLM3 cells that were tranfected with scrambled siRNA or BCORL1 siRNA-1 were subjected to Western blot for BCORL1. *n* = 6; ^*^ *P* < 0.05 by *t* test. B) Transwell migration assays showed that BCORL1 knockdown inhibited cell migration in HCCLM3 cells. As assessed by Transwell invasion assays, HCCLM3 cell invasion was inhibited by BCORL1 knockdown. ^*^ *P* < 0.05 by *t* test; *n* = 3. (TIF 1951 kb) Additional file 2: Figure S2. BCORL1 knockdown does not affect HCC cell proliferation. HCCLM3 and MHCC97H cells that were transfected with scramble siRNA or BCORL1 siRNA were subjected to BrdU incorporation assays. Quantitative data indicated that BCORL1 knockdown did not significantly influence cell proliferation in both HCCLM3 and MHCC97H cells. (TIF 72 kb)

## Abbreviations

AOM: azoxymethane
BCORL1: BCL6 corepressor-like 1
CtBP: C-terminal-binding protein
DMEM: Dulbecco’s modified Eagle medium
DSS: dextran sulfate sodium
ELF4: E74-like factor 4
EMT: Epithelial-mesenchymal transition
HBV: Hepatitis B virus
HCC: Hepatocellular carcinoma
HRP: Horseradish peroxidase
OS: Overall survival
qRT-PCR: Quantitative reverse transcription polymerase chain reaction
RFS: Recurrence-free survival
SDS-PAGE: sodium dodecyl sulfate polyacrylamide gel electrophoresis
SP-IHC: Streptavidin peroxidase conjugate-immunohistochemistry
TNM: Tumor-node-metastasis
UICC/AJCC: International Union Against Cancer/American Joint Committee on Cancer
ZEB1/2: Zinc finger E-box-binding homeobox 1/2
